RETRACTED

# COL10A1-DDR2 axis promotes the progression of pancreatic cancer by regulating MEK/ERK signal transduction

**DOI:** 10.3389/fonc.2022.1049345

**Published:** 2022-11-30

**Authors:** Zhihui Wen, Jingbo Sun, Junjie Luo, Yun Fu, Yue Qiu, Yanyan Li, Yangwei Xu, Hongmei Wu, Qingling Zhang

**Affiliations:** ^1^ Department of Pathology, Guangdong Provincial People’s Hospital, Guangdong Academy of Medical Sciences, Guangzhou, Guangdong, China; ^2^ Department of Pathology, School of Basic Medical Sciences, Southern Medical University, Guangzhou, Guangdong, China; ^3^ Institute of Hematology, Union Hospital, Tongji Medical College, Huazhong University of Science and Technology, Wuhan, China; ^4^ Department of General Surgery, The Third Affiliated Hospital of Southern Medical University, Guangzhou, Guangdong, China

**Keywords:** COL10A1, DDR2, pancreatic cancer, metastasis, EMT

## Abstract

Pancreatic ductal adenocarcinoma (PDAC) is one of the most lethal malignant tumors with a poor prognosis. Type X collagen α 1 chain (COL10A1), a member of the collagen family, is a gene associated with the progression of a variety of human tumors, but the specific function and molecular mechanism of COL10A1 in pancreatic cancer remain unclear. Our study found that COL10A1 is highly expressed in pancreatic cancer cells and tissues, and its high expression is related to poor prognosis and some clinicopathological features, such as tumor size and differentiation. Biological functional experiments showed that overexpression of COL10A1 enhanced the proliferation and migration of PDAC cells. Interestingly, discoid protein domain receptor 2 (DDR2), the receptor of COL10A1, is regulated by COL10A1. We found that the COL10A1-DDR2 axis activates the mitogen-activated protein kinase (MEK)/extracellular signal-regulated kinase (ERK) pathway, which leads to epithelial-mesenchymal transformation (EMT) and accelerates the progression of pancreatic cancer. In summary, COL10A1 regulates PDAC cell proliferation and MEK/ERK signaling pathways by binding to DDR2 to promote migration, invasion and EMT. Our study suggested that COL10A1 might be a critical factor in promoting PDAC progression. More research is needed to confirm COL10A1 as a potential biomarker and therapeutic target for PDAC.

## Introduction

Pancreatic ductal adenocarcinoma (PDAC) is a malignant tumor with high mortality due to its difficulty in early diagnosis, rapid progression, and limited effective therapy. In recent years, morbidity and mortality have increased. Despite improvements in treatment, the overall 5-year survival rate of PDAC remains relatively unchanged (1, 2) and ranked the lowest in the latest cancer statistics in 2022 (3). Notably, drugs based on the molecular pathogenesis of tumors, such as targeted therapies and immune checkpoint inhibitors, have made indelible achievements in the field of cancer immunotherapy (4, 5). However, surgery and chemotherapy remain the current common treatments for PDAC (6). Therefore, it is of great significance to further elucidate the mechanism of PDAC and explore more possible treatments for PDAC.

RETRACTED

Collagen X (collagen type X, COL10) is a homologous trimeric nonfibrillar collagen in the human body that belongs to the collagen family. Type X collagen alpha 1 chain (collagen type X alpha 1 chain, COL10A1) is a specific cleavage fragment of type X collagen (7). COL10A1 consists of an N-terminal signal peptide (amino acids 1-18), noncollagen domain 2 (noncollagenous domain 2, NC2) (amino acids 19-56), triple helix region (amino acids 57-519) and C-terminal noncollagen domain 1 (noncollagenous domain 1, NC1) (amino acids 520-680) (8). The mutation and abnormal expression of COL10A1 are usually accompanied by abnormal chondrocyte hypertrophy, which is related to bone disease and osteoarthritis (9, 10). In recent years, research on the role of COL10A1 in tumors has gradually increased. COL10A1 expression is low in most normal tissues, elevated in many different tumor types (such as colon cancer (11), esophageal cancer (12), gastric cancer (13) and breast cancer (14)) and has been related to the tumor vascular system through immunofluorescence (15). *Tingting Li* et al. found that TGF-β1 could upregulate the expression of COL10A1 through the transcription factor SOX9 in gastric cancer (13), while other studies have shown that COL10A1 is abnormally expressed in colorectal cancer and involved in the progression and EMT process of colorectal cancer (16). The current study found that high expression of COL10A1 in pancreatic cancer is associated with poor prognosis of pancreatic cancer (17). However, the biological function of COL10A1 in PDAC and its molecular mechanisms related to the progression of PDAC are still unknown.

Collagen mainly interacts with cancer cells by directly connecting with cancer cell receptors (18, 19), including integrins, discoid protein domain receptors and tyrosine kinase receptors. It has been shown that collagen in the microenvironment promotes tumor growth in colorectal cancer cells by activating the PI3K/AKT signaling pathway through the membrane surface receptor α2 β1 (20). Remodeled COLI(Type I collagen) affects the invasion of ovarian cancer cells by mediating the integrin PTEN/PI3K/AKT signal transduction pathway (21). Discoidin domain receptor (DDR) is a subfamily of tyrosine kinases (RTKs) that are divided into homologous DDR1 and DDR2 receptors (22). DDR is the only RTK that specifically binds to and is activated by collagen. Studies have shown that the interaction between COLI and DDR1 affects the protein tyrosine kinase associated with focal adhesion kinase (FAK), resulting in the upregulation of N-cadherin in PDAC cells, which induces EMT (23); it was further reported that COLI activates DDR2 and stimulates ERK2 in an Src-dependent manner (24). Notably, COL11A1 binds to α1β1 integrin and DDR2 to activate the Src-phosphatidylinositol 3-kinase (PI3K)/AKT-NFκB pathway to induce the expression of three cisplatin-induced apoptosis inhibitors in ovarian cancer (25). Previous studies have found that type X collagen is mainly the ligand of DDR2 (26), and DDR2 has been shown to promote the progression and metastasis of many cancers (26). However, the interaction between COL10A1 and DDR2 has not been reported to affect PDAC progression.

RETRACTED

In this study, we aimed to probe the function and mechanism of COL10A1 in regulating PDAC progression. Based on a series of *in vitro* and *in vivo* experiments, we first proved that overexpression of COL10A1 promoted the proliferation and migration of PDAC cells. Next, we demonstrated that COL10A1-DDR2 axis-induced EMT was dependent on MEK/ERK pathway activation. These results deepen our understanding of PDAC progression and may provide new therapeutic strategies for PDAC patients.

## Results

### COL10A1 is upregulated in PDAC and predicts poor prognosis

Analysis of the GEO (GSE15471) database revealed that COL10A1 was differentially expressed in pancreatic cancer versus normal tissue (**Figure 1A**) and that COL10A1 was highly expressed in tumor tissues compared with normal tissues of PDAC patients in the GEPIA dataset (**Figure 1B** and **Supplementary Figure 1A**). To investigate the role of COL10A1 in PDAC, we performed IHC staining of COL10A1 using 64 cases of PDAC and matched adjacent normal pancreatic tissue samples (**Figure 1C**). The level of COL10A1 expression was significantly higher in PDAC than in normal tissues (**Figure 1D**). High expression of COL10A1 was detected in 81.3% (52/64) of PDAC tissue samples and only 14.1% (9/64) of normal pancreatic tissue samples (**Figure 1E**). In addition, according to the AJCC 8th edition pancreatic cancer staging criteria, the frequencies of high COL10A1 expression were T1, 55.6% (5/9); T2, 81.8% (27/33); T3, 90.9% (20/22); and T4, 0 (0), indicating that COL10A1 expression was positively correlated with the tumor T stage. High expression of COL10A1 was observed in 71.4% (25/35) and 93.1% (27/29) of well-moderately and poorly differentiated tumors, respectively (**Figure 1F** and **Table 1**), suggesting that COL10A1 expression is negatively correlated with PDAC differentiation. Moreover, the overexpression of COL10A1 was closely correlated with shorter overall survival of PDAC patients (**Figure 1G** and **Supplementary Figure 1B**). Subsequently, the endogenous expression of COL10A1 was analyzed in four PDAC cell lines (PANC-1, SW1990, BXPC-3, and CFPAC-1) and the normal human pancreatic epithelial cell line HPDE6-C7 (**Figure 1H**), where COL10A1 was found to be more highly expressed in PDAC cell lines than in HPDE6-C7.

RETRACTED

**Figure 1:** COL10A1 is up-regulated in PDAC and predicts poor prognosis. **(A)** GEO database (GSE15471) analysis to screen for genes that differ more significantly in pancreatic cancer versus normal tissue. **(B)** The GEPIA dataset showed that COL10A1 was highly expressed in a variety of tumors, and that COL10A1 expression was significantly higher in pancreatic cancer than in normal tissues. **(C)** IHC staining of COL10A1 in PDAC and normal pancreatic tissues. The scale bar at 200× magnification represents 20 µm. The scale bar at 400× magnification represents 50 µm. **(D)** COL10A1 IHC scores were differentially expressed between the normal and tumor groups. n = 64. Two-tailed Student’s t-test. **(E)** Percentage of COL10A1 IHC in PDAC and matched adjacent normal pancreatic tissues. n = 64. Chi-square test. **(F)** IHC staining analysis of COL10A1 expression in PDAC tissues with T classification and different differentiation characteristics. n = 64. Chi-square test. **(G)** Kaplan-Meier survival analysis of PDAC patients with high or low COL10A1 expression based on IHC data. **(H)** COL10A1 protein levels were detected in PDAC cell lines and one normal pancreatic ductal epithelial cell by western blot analysis. **(I, J)** COL10A1 expression was detected using western blot and RT-PCR by transfecting PDAC cell lines with COL10A1 shRNA and COL10A1-sense plasmids. *P < 0.05, **P < 0.01, ***P < 0.001, ****P < 0.0001.

**Table 1:** Clinical characteristics of PDAC patients with low COL10A1 expression and high COL10A1 expression.

Characteristics	n	COL10A1 expression		*P*
		Low (%)	High (%)
**Age(y)**				
≥60	35	8 (22.9%)	27 (77.1%)	0.355
<60	29	4 (13.8%)	25 (86.2%)	
**Gender**				
Male	35	4 (11.4%)	31 (88.6%)	0.99
Female	29	8 (27.6%)	21 (72.4%)	
**clinical stage**				
I	32	7 (21.9%)	25 (78.1%)	0.442
II	29	5 (17.2%)	24 (82.8%)	
III	0	0	0	
IV	3	0	3 (100%)	
**T classification**				
T1	9	4 (44.4%)	5 (55.6%)	0.042
T2	33	6 (18.2%)	27 (81.8%)	
T3	22	2 (9.1%)	20 (90.9%)	
T4	0	0	0	
**N classification**				
N0	41	7 (17.1%)	34 (82.9%)	0.646
N1	23	5 (21.7%)	18 (78.3%)	
**Metastasis**				
No	61	12 (19.7%)	49 (80.3%)	0.394
Yes	3	0	3 (100%)	
**Histological type**				
Well/Moderately	35	10 (28.6%)	25 (71.4%)	0.027
Poorly	29	2 (6.9%)	27 (93.1%)	

Taken together, these results suggested that the overexpression of COL10A1 is associated with advanced PDAC progression and could be used as a prognostic marker in PDAC. In summary, these results demonstrated that COL10A1 overexpression is highly correlated with poor differentiation, tumor T stage, and poor prognosis in PDAC.

RETRACTED

### COL10A1 promotes PDAC proliferation and migration

To investigate the function of COL10A1 in the progression of PDAC, cells with low (PANC-1 and CFPAC-1) and high (SW1990 and BXPC-3) COL10A1 expression were selected to establish COL10A1 knockdown (SW1990.shCOL and BXPC-3.shCOL) (**Figure 1I**) and COL10A1 overexpression (PANC-1. COL and CFPAC-1. COL) (**Figure 1J**) cell lines, respectively. We selected the most efficient siRNA sequences to package the lentivirus, thus constructing the COL10A1 knockdown group (SW1990.shCOL and BXPC-3.shCOL) (**Supplementary Figures 2A, B**). The cell counting kit-8 (CCK8) and colony formation assay results showed that the proliferation and colony formation ability of SW1990.shCOL and BXPC-3.shCOL cells were significantly inhibited compared with those of the control groups (**Figures 2A, C, D** and **Supplementary Figures 3A, C, D**), while these abilities were significantly increased in PANC-1.COL and CFPAC-1.COL cells (**Figures 2B, C, E** and **Supplementary Figures 3B, C, E**). Transwell and wound healing assay results showed that the migration abilities of the COL10A1 overexpression cells were significantly higher than those of the control cells (**Figures 2G–K** and **Supplementary Figures 3G–I, K**), whereas they were decreased in the COL10A1 knockdown cells (**Figures 2F, H–J** and **Supplementary Figures 3F, H–J**).

**Figure 2:** COL10A1 promotes PDAC proliferation and migration *in vitro*. **(A-C)** Colony formation assays to determine the effect of COL10A1 on the proliferation of PDAC cells. **(D, E)** Cell proliferation analyses of the PDAC cells. **(F-H)** Migration ability of cells was tested using wound healing assay. **(I-K)** Transwell assays detect changes in cell migration after knockdown and overexpression of COL10A1. *P < 0.05, **P < 0.01, ***P < 0.001, ****P < 0.0001.

To further investigate the functions of COL10A1 *in vivo*, subcutaneous tumor models were established to assess tumor growth. Tumors grew faster in the PANC-1.COL group than in the PANC-1.Veh group. In addition, the COL10A1 knockdown groups were reduced accordingly (**Figures 3A-D**). The Ki-67 index was higher in PANC-1.COL tumors and lower in BXPC-3.shCOL tumors compared to the controls (**Figures 3E, F**). The orthotopic mouse tumor model observations showed that the average tumor volume was smaller in the BXPC-3.shCOL group than in the BXPC-3.Scr group (**Figures 3G, H**). The number of liver metastases was lower in the BXPC-3.shCOL group than in the BXPC-3.Scr group (**Figures 3G, I**). No metastasis was observed in other organs within the investigated period. These results suggest that COL10A1 can significantly promote tumor formation and metastasis in the orthotopic mouse tumor model. Following this, the *in vitro* and *in vivo* results indicated that COL10A1 functions as a tumor metastasis oncogene that can dramatically promote PDAC progression and liver metastasis.

RETRACTED

**Figure 3:** COL10A1 promotes PDAC proliferation and migration *in vivo*. **(A, B)** Images of gross PDAC subcutaneous xenograft tumor models formed by the indicated cell lines. **(C, D)** tumor volume and weight analyses for the subcutaneous xenograft tumor. Means ± SD are provided (n=5). **(E)** Representative images of H&E staining and ki67, COL10A1 IHC staining of tumors from subcutaneous xenograft tumor models. Scale bars, 50 μm. **(F)** The percentage of positively stained Ki-67 cells in subcutaneous tumors. **(G)** Representative images of gross and H&E staining in PDAC orthotopic models formed by the indicated cell lines. Means ± SD are provided (n=9). Scale bars, 50 μm. **(H)** tumor volume analyses of the PDAC primary tumors in PDAC orthotopic models. **(I)** The metastatic nodules in the livers per group were counted. *P < 0.05, **P < 0.01, ***P < 0.001, ****P < 0.0001.

### COL10A1 regulates DDR2 expression in PDAC cells

DDRs are the only RTKs that can specifically bind to and be activated by different types of collagen. The discoidal domain receptors are divided into homologous DDR1 and DDR2 receptors. The activation of each receptor responds to the unique signaling pathway of collagen and triggers different cellular responses (27). Previous findings have suggested that DDR2 binds preferentially to collagen II and collagen X (26). Using GEPIA and cBioPortal tools for gene coexpression analysis, we found a significant correlation between the mRNA levels of COL10A1 and DDR2 in PDAC tissues, and DDR2 was also highly expressed in PDAC (**Supplementary Figures 4A, B**). Western blotting was performed to detect the expression of DDR1 and DDR2 in PDAC, and we found that DDR2 expression levels were similar to COL10A1, in that they were highly expressed in SW1990 and BXPC3 cells and less expressed in CFPAC-1 and PANC cells (**Supplementary Figure 4C**). Moreover, COL10A1 upregulated the mRNA level of DDR2 in PDAC cells (**Supplementary Figure 4D**). And COL10A1 upregulated the protein level of DDR2 and phosphorylated DDR2 (p-DDR2) in PANC-1 and CFPAC-1 cells, while the inhibition of COL10A1 reduced this phenotype in SW1990 and BXPC-3 cells (**Figure 4A**). To investigate the role of DDR2 in PDAC, we performed IHC staining of DDR2 using 30 cases of PDAC and matched adjacent normal pancreatic tissue samples (**Figure 4B**). The level of DDR2 expression was significantly higher in PDAC than that in normal tissues (**Figure 4C**). Statistical analysis of clinical characteristics showed that high DDR2 expression was highly correlated with lymph node metastasis (*p*=0.037) and positively correlated with clinical stage at a trend close to significance (*p*=0.082, **Supplementary Table 1**). In addition, the level of DDR2 expression was positively correlated with COL10A1 in PDAC (**Figure 4D**). Therefore, we speculated that the COL10A1-DDR2 axis is activated in PDAC cells. IF staining results verified that COL10A1 and DDR2 were colocalized in PDAC cells (**Figure 4E**). Furthermore, Co-IP assays were performed and confirmed our hypothesis that there was an interaction between COL10A1 and DDR2 in PANC-1 and HEK293T cells (**Figures 4F, G**). These results demonstrated that COL10A1 overexpression distinctly enhances DDR2 levels and that COL10A1 exerts a positive moderating effect on DDR2 activation.

RETRACTED

**Figure 4:** COL10A1 regulates DDR2 expression in PDAC cells. **(A)** Western blot results showed the effect of COL10A1 on DDR2 and P-DDR2 protein levels. **(B)** IHC staining of DDR2 in PDAC and normal pancreatic tissues. The scale bar at 200× magnification represents 20 µm. The scale bar at 400× magnification represents 50 µm. **(C)** DDR2 IHC scores were differentially expressed between the normal and tumor groups. n = 30. Two-tailed Student’s t-test. **(D)** Pearson correlation analysis was conducted to analyze the relation between COL10A1 and DDR2 in 30 PDAC tissues. **(E)** Co-localization of COL10A1 and DDR2 in PDAC cells detected by immunofluorescence. **(F, G)** The detection of the interaction between COL10A1 and DDR2 by Co-IP. ***P<0.001.

### COL10A1 facilitates the malignant biological behavior of PDAC cells through DDR2

We verified that there is indeed a regulatory relationship between COL10A1 and DDR2 and then further investigated the role of DDR2 in the biological function of PDAC. CCK-8 and colony formation assays were used to detect changes in the proliferation ability of the Scramble group, shCOL10A1 group, and shCOL10A1+DDR2 group in SW1990 and BXPC-3 cell lines. The results showed that the proliferation ability of the shCOL10A1 group was significantly reduced compared to that of the Scramble group, while the shCOL10A1+DDR2 group significantly reversed this inhibitory effect (**Figures 5A, B**). Likewise, Transwell and wound healing assays showed that DDR2 overexpression dramatically reversed the inhibitory effects of COL10A1 knockdown on migration (**Figures 5C-I**).

RETRACTED

**Figure 5:** COL10A1 facilitates the malignant biological behavior of PDAC cells through DDR2. **(A)** Effect of DDR2 overexpression on the proliferative capacity of SW1990, BXPC cells after disruption of COL10A1 using clone formation assay. **(B)** Effects of shCOL and shCOL10A1+DDR2 on the proliferation ability of SW1990 and BXPC-3 cells by CCK8 assay. **(C-F)** Effects of shCOL and shCOL10A1+DDR2 on the migration ability of SW1990 and BXPC-3 cells by wound healing assays. Scale bar, 50 µm. **(G-I)** Effects of shCOL and shCOL10A1+DDR2 on the migration ability of SW1990 and BXPC-3 cells by transwell assays. Scale bar, 50 µm. *P < 0.05, **P < 0.01, ****P < 0.0001. ns, no significance.

Taken together, these findings suggest that COL10A1 promotes the proliferation and migration ability of PDAC cell lines *in vitro* by promoting the expression of DDR2.

### COL10A1-DDR2 induces PDAC cell EMT

Previous studies of DDR2 have emphasized that the upregulation of DDR2 plays a crucial role in inducing the EMT pathway (28, 29). Eighteen tumor tissues each were divided into groups of low and high expression of COL10A1, and the GSEA pathway enrichment results showed that high COL10A1 expression was associated with EMT and the TGF-β signaling pathway (**Figure 6A**). To assess whether COL10A1 activation of DDR2 induced EMT in PDAC cells, we first observed the morphology of cells with COL10A1 overexpression or knock down under a microscope. COL10A1 overexpression in PANC-1 cells resulted in a spindle-shaped and fibroblastic-like phenotype. Their control cells, on the other hand, had relatively tight cell-cell adhesion, and the cells displayed a round, flat or mixed morphology with a short cytoplasmic extension; the opposite effect was obtained for BXPC-3 cells with COL10A1 knockdown (**Supplementary Figure 5A**). Next, IF was used to detect changes in EMT-related markers. Consistent with our hypothesis, the expression levels of the epithelial marker E-cadherin were distinctly decreased, and the mesenchymal markers N-cadherin and Vimentin were dramatically increased in the COL10A1 overexpression group (**Figure 6B**). The western blot results further revealed that overexpression of COL10A1 decreased the expression levels of E-cadherin, and dramatically increased the expression levels of N-cadherin, Vimentin and Snail. In contrast, knockdown of COL10A1 achieved the opposite effect (**Figure 6C** and **Supplementary Figure 5B**). Furthermore, these inhibitory effects of COL10A1 knockdown were rescued upon DDR2 overexpression (**Figure 6D**). These results suggested that COL10A1 promotes the activation of DDR2 and further induces EMT in PDAC cells.

RETRACTED

**Figure 6:** COL10A1-DDR2 axis promotes EMT in PDAC cells through activation of MEK/ERK pathway. **(A)** GSEA validated EMT-related pathways in high COL10A1 expression PDAC cohorts of GSE15471 dataset. **(B)** The effect of COL10A1 on the expressions of EMT signaling proteins by Immunofluorescence. **(C)** The effect of COL10A1 and DDR2 on the expressions of EMT signaling proteins by Western blot. **(D)** Western blot detection of the effect of overexpression of DDR2 on protein expression changes in the EMT pathway induced by interference with COL10A1. **(E)** Western blot analyses of MEK/ERK pathway proteins in the indicated cells. **(F)** The protein expression of EMT pathway was detected by western blot in PDAC cells after treated with ERK inhibitor SCH772984. **(G)** H&E staining and IHC staining of COL10A1, DDR2, P-ERK, E-cadherin, N-cadherin and Vimentin in PDAC orthotopic models. Scale bars, 20 μm.

### The COL10A1-DDR2 axis promotes EMT in PDAC cells through activation of the MEK/ERK pathway

ERK activation is crucial for SNAIL1 stability and EMT induction (29), and we further explored the molecular mechanisms induced by COL10A1 and DDR2. The results showed that, compared to the control cells, the phosphorylation levels of ERK and MEK were upregulated in both PANC-1.COL and CFPAC-1.COL cells but downregulated in BXPC-3.shCOL and SW1990.shCOL cells (**Figure 6E** and **Supplementary Figure 5C**). These results indicated that COL10A1-DDR2 activates MEK/ERK pathway activity.

To confirm whether the COL10A1-DDR2 axis induces the EMT process in PDAC cells by activating the MEK/ERK pathway, we used the ERK inhibitor SCH772984 on PANC-1.COL10A1 and CFPAC-1.COL10A1 cells. Western blot analysis was utilized to determine the protein levels of p-ERK and EMT pathway markers (E-cadherin, N-cadherin, Vimentin and Snail) in the treatment and control cells (**Figure 6F**). The IHC assay of PDAC orthotopic mouse tumors revealed that knockdown of COL10A1 enhanced the expression of E-cadherin (epithelial marker) and decreased the expression of N-cadherin and Vimentin (mesenchymal marker). We also found that the expression of p-ERK was significantly reduced (**Figure 6G**). In conclusion, these results suggested that the EMT process can be triggered by MEK/ERK in pancreatic cancer (**Figure 7**).

**Figure 7:** Model: COL10A1 activated the MEK/ERK signaling pathway of pancreatic cancer cells and promoted the EMT of pancreatic cancer cells through a DDR2-dependent pathway.

RETRACTED

## Discussion

Previous evidence has indicated that collagen is a major component of the tumor microenvironment, serving as a dependency and scaffold for cell growth and inducing epithelial cell proliferation, differentiation and migration (30). PDAC is among the deadliest human malignancies, and a hallmark of the disease is a distinctive collagen-rich fibrotic extracellular matrix (31). Increased fibrosis due to collagen deposition and metabolic dysregulation can promote tumor development and invasion (32, 33). COL10A1 is a member of the collagen family, and current studies on COL10A1 have found that it is highly expressed in most tumor tissues, and its elevated expression is associated with tumor angiogenesis (27, 34). However, the biological functions and mechanisms of COL10A1 in PDAC have not been reported. In our study, the high expression of COL10A1 in PDAC tissues was verified; analysis of clinicopathological consequences showed that COL10A1 was positively correlated with tumor T stage, negatively correlated with the degree of differentiation, and associated with poor prognosis in pancreatic cancer patients. Furthermore, functional experiments indicated that COL10A1 overexpression promotes PDAC cell proliferation and migration both *in vitro* and *in vivo*. These results confirmed that COL10A1 is a tumor oncogene in PDAC and that the overexpression of COL10A1 is partially responsible for PDAC progression.

Studies on collagen and tumor orientation have found that cancer cells can regulate collagen biosynthesis through mutated genes, transcription factors, signaling pathways, and receptors (30, 31). In addition, collagen can also influence the behavior of tumor cells through integrins, discoidal protein structural domain receptors, tyrosine kinase receptors, and several signaling pathways (32). Several studies have shown that collagen in the tumor microenvironment promotes the growth of colorectal cancer cells by activating the PI3K/AKT signaling pathway through the membrane surface receptor integral protein α2β1 (20). Remodeled collagen I (COLI) promotes ovarian cancer cell invasion by mediating the integral protein PTEN/PI3K/AKT signaling pathway (21). DDR2 belongs to a subfamily of receptor tyrosine kinases (RTKs) and regulates tumor growth and invasion by binding to fibrillar and nonfibrillar collagen activation (35). DDR2, an RTK, is upregulated in a variety of cancer cells and is associated with poor prognosis in many cancer types (33, 36). The DDRs have distinct preferences for certain types of collagens. DDR2 seems to preferentially bind collagen II and collagen X (26). Our findings suggested that COL10A1 promotes the proliferation and migratory capacity of pancreatic cancer cells *in vitro* by promoting DDR2 expression and activation.

RETRACTED

Accumulating evidence suggests that a unique set of RTKs, known as discoidin domain receptors, play a role in cancer progression by regulating the interactions of tumor cells with their surrounding collagen matrix (27, 34). Upon binding to collagen, the DDR undergoes self-phosphorylation with very slow and sustained kinetics (37). Hence, DDRs are part of the signaling networks that convert extracellular matrix information and thus serve as key regulators of cell-matrix interactions. Under physiological conditions, DDRs control cell and tissue homeostasis by acting as collagen sensors, transducing signals that regulate cell polarity, tissue morphogenesis, and cell differentiation (38, 39). In cancer, DDRs are hijacked by tumor cells to disrupt normal cell-matrix communication and initiate promigratory and proinvasive programs (38, 39). In tumor-related studies, DDR2 is upregulated in a variety of cancer cells, and DDR2 is a major regulator of EMT, promoting the EMT process in cancers such as breast cancer (40, 41), liver cancer (28), and thyroid cancer (29). ERK signaling is a ubiquitous signal transduction pathway that regulates important cellular processes, such as proliferation, migration and invasion (42, 43). A growing body of evidence has shown that activation of ERK contributes to the development of many types of cancer. Zhong Liang et al. found that upregulation of DDR2 induced EMT through activation of the ERK2/Snail1 signaling pathway and promoted cell migration and invasion of papillary thyroid cancer cells, demonstrating that ERK activation is essential for Snail1 stabilization and EMT induction (29). To investigate the molecular mechanism of COL10A1 binding to DDR2 that promotes the proliferation and metastasis of pancreatic cancer, we first observed the cell morphology and examined the relevant indicators of EMT. It was found that COL10A1 activation of DDR2 resulted in fibroblast-like cells with reduced E-cadherin expression and increased expression of Vimentin, Snail and N-cadherin. In contrast, cells after COL10A1 knockdown appeared oblate, and EMT processes were inhibited. In our study, we further indicated that COL10A1-DDR2 axis-induced EMT was dependent on MEK/ERK pathway activation.

In this study, we identified a key molecular biomarker, COL10A1, whose expression was elevated in PDAC. COL10A1 enhances the proliferation and migration of PDAC cells by promoting DDR2 expression and activation. Mechanistically, COL10A1 accelerated the proliferation and metastasis of pancreatic cancer by activating the MEK/ERK signaling pathway and promoting EMT in PDAC cells through a DDR2-dependent pathway (**Figure 7**). Clinically, COL10A1 correlates with PDAC tumor stage and differentiation and can be a poor prognostic factor for PDAC. Patients with PDAC with high COL10A1 expression had shorter survival. In conclusion, these findings point to a new mechanism of COL10A1 involvement in PDAC progression. Many studies have shown the potential of DDR inhibition as a novel therapeutic strategy (34, 44, 45). DDR2 serves as a major target for enhancing the response to anti-PD-1 immunotherapy, and this combination therapy has been validated in a variety of tumors (5, 46). Our study elucidated the important role of the COL10A1-DDR2 axis in PDAC. The design of inhibitors targeting the COL10A1-DDR2 axis may be a novel target for PDAC-targeted combined immunotherapy. This provides a new option for the diagnosis, treatment and prognosis of clinical PDAC.

RETRACTED

There are several deficiencies as well as limitations of our study. First, we should have validated DDR2 expression and the relationship with COL10A1 in more clinical samples, which may have greater clinical significance. Second, further studies exploring the specific mechanisms of how COL10A1 induces DDR2 expression and phosphorylation and subsequent studies on DDR2 inhibitors would be therapeutically helpful.

## Materials and methods

### Gene set enrichment analysis

Gene set enrichment analysis (GSEA) was used to identify the signaling pathways that correlated with gene expression. To probe the biological mechanisms using GSEA software v4.2.3 (Broad Institute, MIT, Cambridge, MA, USA), a 54675 (gene)×36 (samples) expression matrix was employed. The predefined gene set ‘HALLMARK. Gmt’ is one of 7 major collections from the Molecular Signatures Database (MSigDB). Gene sets were considered significantly enriched at predefined p values and FDR < 0.25, and NES was calculated as the primary GSEA statistic.

### Tissue specimens and cell culture

We collected a cohort of 64 paraffin-embedded specimens from patients with resectable primary PDAC who underwent pancreaticoduodenectomy at Nanfang Hospital, Southern Medical University from 2016 to 2018. Prior patient consent and approval were obtained from the Institutional Research Ethics Committee. PDAC cell lines, including SW1990, PANC-1, BXPC-3, and CFPAC-1, and the normal human pancreatic duct epithelium cell line HPDE6-c7 were provided by Shanghai Cell Bank (Chinese Academy of Sciences, Shanghai, China). All cell lines (8 × 10^5^ cells/plate) were seeded in Dulbecco’s modified Eagle’s medium (DMEM) (HyClone, Logan, UT, USA) with 10% fetal bovine serum (FBS, Gibco, Brazil) at 37°C in a 5% CO_2_ incubator.

RETRACTED

### Cell transfection

The siRNAs for COL10A1 interference were constructed and generated by Genechem (Shanghai, China). The COL10A1 overexpression lentivirus (LV-COL10A1), overexpression control lentivirus (Vector), shCOL10A1 stable expression lentivirus (shCOL10A1: CCGGGCTTCCCAATGCCGAGTCAAACTCGAGTTTGACTCGGCATTGGGAAGCTTTTT), and control stable expression lentivirus (Scramble) were all synthesized and purchased from GeneChem Co., Ltd. (Shanghai, China). The COL10A1 overexpression plasmid carries the FLAG tag (CMV enhancer-MCS-3flag-polyA-EF1A-zsGreen-sv40-puromycin), and the DDR2 overexpression plasmid carries the HA tag (CMV-MCS-IRES-mCherry-SV40-Neomycin) from GeneChem Co., Ltd. (Shanghai, China).

The human PDAC cell lines PANC-1 and CFPAC-1 were transfected with LV‐COL10A1 or vector, while the cell lines SW1990 and BXPC-3 were transfected with shCOL10A1 or scramble. HEK293T and PANC-1 cells were transfected with COL-Flag or DDR-HA. PDAC cell lines were seeded into 24‐well plates using HiTransG P (20 μl/well, GeneChem, Shanghai, China). After being transfected for 48 h, the cells were collected and used for the following experiments. The efficiency of infection could be assessed through Western blotting after puromycin-selected or neomycin-selected cells for 1-2 weeks.

### RNA extraction and quantitative reverse transcription PCR

Total RNA was extracted from PDAC cell lines with RNAiso-Plus (TAKARA, Dalian, China). Single-stranded cDNA was then synthesized from 1 μg extracted mRNA using an RT−PCR cDNA synthesis kit (TAKARA, Dalian, China) according to the manufacturer’s instructions. RT−PCR was performed using an Applied Biosystems 7500 Sequence Detection system with iQ™ SYBR green supermix (Bio-Rad Laboratories, Hercules, CA, USA). The primer sequences used in this study were as follows: COL10A1 forward primer 5′‐TGACGAGACCAAGAACTGCC‐3′ and reverse primer 5′‐GCACCATCATTTCCACGAGC‐3′; β‐actin forward primer 5′‐GCTCGTCGTCGACAACGGCTC‐3′ and reverse primer 5′‐CAAACATGATCTGGGTCATCTTCTC‐3′.

### Immunohistochemistry

The paraffin-embedded sections were stepwise dewaxed from xylene and gradient ethanol to water, and IHC staining was performed according to the protocol. IHC staining was performed with heat-induced antigen retrieval, followed by incubation in primary antibodies overnight at 4°C, secondary antibody (EnVision/HRP kit, DAKO) for 30 min at RT (room temperature) and substrate-chromogen solution (DAB detection kit, DAKO) for 5 min at RT, with hematoxylin counterstain for 10 s. At each step, the slides were washed in PBS three times for 5 min. Two pathologists independently evaluated and scored the sections, and the IHC score was estimated as a sum of the staining intensity and percentage of positive tumor cells. Briefly, the staining intensity was scaled from 0–3 (0: negative, 1: weak positive, 2: moderate positive, 3: strong positive), and the percentage of positive cell staining was scored from 0–4 (0: ≤2%, 1: 2%–10%, 2: 10%–50%, 3: 50%–80%, 4: 80%–100%). The final staining was summed by intensity and percentage as 0–12. Then, the scores were adapted to a 4-point IRS: 0–1 (−), 2–3 (+), 4–8 (++), and 9–12 (+++). Finally, we set −~+ as COL10A1 Low expression and ++~+++ as COL10A1 High expression. The clinicopathological significance of the IHC data was analyzed by Chi-square analysis. IHC staining and statistics were performed blindly.

RETRACTED

### Western blot analysis

The proteins were dissociated and separated by SDS/PAGE and then transferred to PVDF membranes, which were incubated with primary antibodies. The following primary antibodies were used: DDR2, 1:1000, ABclonal; p-DDR2, 1:1000, R&D; COL10A1, 1:1000, BOSTER; β-actin, 1:1000, Abcam; E-cadherin, N-cadherin, Vimentin, Snail, MEK, p-MEK, ERK, and p-ERK, 1:1000 (Cell Signaling Technology). Subsequently, the membranes were incubated with horseradish peroxidase‐conjugated secondary antibodies for 60 min. Signals were then visualized by an enhanced chemiluminescence kit. The grayscale value of each band was measured by ImageJ and compared with the corresponding internal parameters.

### Wound healing assay

For the wound healing assay, pretreated cells were seeded into 6-well plates and cultured until 100% confluent. The monolayer was wounded using a 10 µl pipette tip, and cells were then washed to remove cell debris and continuously cultured in DMEM culture medium with 1% FBS. Images were taken at 0 and 24 h after scratching.

### Transwell assay

In total, 1 × 10^5^ cells were seeded into the upper chamber (BD Biosciences, San Jose, CA, USA) with a serum-free medium. Medium (10% FBS, Invitrogen) was added to the lower chamber, and the medium served as a chemoattractant. After incubation at 37°C and 5% CO_2_ for 48 h, the chambers were placed in 4% paraformaldehyde for 30 min and then stained with 2% crystal violet for 30 min. The numbers of migrated cells were calculated in five random fields per well.

### Cell counting kit 8 assay and clone formation assay

For CCK8 assays, 2 × 10^3^ cells were seeded into each well of a 96-well plate in triplicate. After incubating for the indicated time, 10 μl of CCK-8 buffer (Dojindo, Japan) was added to each well and incubated for 2 h at 37°C. Then, the absorbance data (OD value) at a wavelength of 450 nm were collected for cell viability analysis. This experiment was repeated three times.

RETRACTED

For colony formation assays, cells were plated in 6-well plates (300 cells/well) and cultured for 2 weeks until the appearance of cell colonies. The colonies were fixed and stained with hematoxylin, and those containing more than 50 cells were counted for further statistical analysis. Each experiment was repeated three times.

### Coimmunoprecipitation analysis

Co-IP assays used antibodies specific for anti-HA (Proteintech; 51064-2-AP) and anti-FLAG (CST; 14793S). Briefly, cells were washed with ice-cold PBS and lysed in cold RIPA buffer. Cellular lysates were incubated with antibody overnight, followed by incubation with protein A/G-sepharose beads (Santa Cruz Biotechnology) for 12 h, centrifugation at 2500 g, and three washes with ice-cold lysis buffer. The immunoprecipitated proteins were eluted by denaturation in Laemmli buffer at 95°C for 10 min and then detected by western blotting.

### *In vivo* animal model and growth and metastasis assays

BALB/c-nu/nu nude mice (3-4 weeks old) were provided by the Experimental Animal Center of Southern Medical University and certified by Guangdong Provincial Science Bureau. PANC-1 cells stably overexpressing COL10A1 lentivirus (2 × 10^6^) and control cells (5 mice in each group) or BXPC-3 cells with stable COL10A1 knockdown and control cells (5 mice in each group) were injected subcutaneously into the left and right hind legs of mice. A digital caliper was used to estimate the tumor volume (volume = (length × width^2^)/2) from two vertical axes every three days, and a general picture of the tumor was taken. The primary tumor was surgically resected, dehydrated, fixed, embedded in paraffin, and sectioned. The sections were stained with haematoxylin-eosin and observed under a microscope.

Orthotopic PDAC mouse models were established in 4- to 5-week-old BALB/c nude mice. Nude mice were first anaesthetized with pentobarbital (70 μg/kg). The mouse spleen was then positioned, a small incision was made to expose the spleen, and the pancreas attached to the end of the spleen was spread to position the tail of the pancreas. Then, 100 µL (1 × 10^6^ cells) of cells was injected into the tail of the pancreas, the spleen was reset with the pancreas, an appropriate amount of penicillin was injected into the abdominal cavity, and the incision was sutured. The nude mice were sacrificed after approximately 3 weeks, the *in situ* tumor formation in the pancreas and tumor metastasis in each organ were observed, and the tumors were measured and fixed for further study. A digital caliper was used to estimate the primary tumor volume (volume = (length × width^2^)/2).

RETRACTED

### Immunofluorescence

The cells were fixed with 4% paraformaldehyde for 15 min, washed three times, washed three times with PBS and blocked with 10% fetal bovine serum for 30 min. The cells were incubated with primary antibodies at 4°C overnight, after which they were incubated with red goat anti-rabbit antibody (Proteintech, Chicago, IL) for 1 h at RT. The following primary antibodies were used: DDR2, 1:200 (ABclonal); COL10A1, 1:200 (BOSTER); E-cadherin, N-cadherin, Vimentin, 1:200 (Cell Signaling Technology). Subsequently, the cells were restained with 4-amino-6-diamino-2-phenylindole (DAPI, Sigma), and images were captured using an Olympus FV1000 confocal laser scanning microscope (Olympus USA, NY, USA) and a Karl Zeiss inverted laser confocal microscope (LSM 880 with Airyscan, Germany).

### Statistical analysis

Statistical analyses were performed using Prism 8.0 (La Jolla, CA, USA). Student’s t test and one-way analysis of variance (ANOVA) were used to evaluate the significance of the differences among groups. Each experiment was performed at least three times. All data are presented as the means ± standard deviations (SD).

## Data availability statement

The original contributions presented in the study are included in the article/**Supplementary Material**. Further inquiries can be directed to the corresponding author.

## Ethics statement

The studies involving human participants were reviewed and approved by the Institutional Research Ethics Committee. The patients/participants provided their written informed consent to participate in this study. The animal study was reviewed and approved by the Institutional Animal Care and Use Committee of Southern Medical University.

## Author contributions

QZ led the study design and supervised this work. ZW and JS prepared the manuscript and analyzed the data. JS helped with the revising of the manuscript. ZW, YF, YQ, and YL performed the experiments. JS, JL, HW, and YX gave assistance in collecting tissue samples and animal experiments. ZW and JS contributed equally to this work. All authors contributed to the article and approved the submitted version.

## Funding

This project was supported by grants of the National Natural Science Foundation of China (QZ, 81772918, 8197227 and 82173033; YX, 82102712); China Postdoctoral Science Foundation (YX, 2021M690751); Key-Area Research and Development Program of Guangdong Province (2021B0101420005) and High-level Hospital Construction Project (QZ, DFJHBF202108).

## Conflict of interest

The authors declare that the research was conducted in the absence of any commercial or financial relationships that could be construed as a potential conflict of interest.

RETRACTED

## Publisher’s note

All claims expressed in this article are solely those of the authors and do not necessarily represent those of their affiliated organizations, or those of the publisher, the editors and the reviewers. Any product that may be evaluated in this article, or claim that may be made by its manufacturer, is not guaranteed or endorsed by the publisher.

## References

[1] NeoptolemosJPKleeffJMichlPCostelloEGreenhalfWPalmerDH. Therapeutic developments in pancreatic cancer: current and future perspectives. Nat Rev Gastroenterol Hepatol (2018) 15(6):333–48. doi: 10.1038/s41575-018-0005-x 29717230

[2] HaeberleLEspositoI. Pathology of pancreatic cancer. Transl Gastroenterol Hepatol (2019) 4:50. doi: 10.21037/tgh.2019.06.02 31304427PMC6624347

[3] SiegelRLMillerKDFuchsHEJemalA.. Cancer statistics, 2022. CA Cancer J Clin (2022) 72(1):7–33. doi: 10.3322/caac.21708 35020204

[4] BagchiSYuanREnglemanEG. Immune checkpoint inhibitors for the treatment of cancer: Clinical impact and mechanisms of response and resistance. Annu Rev Pathol (2021) 16:223–49. doi: 10.1146/annurev-pathol-042020-042741 33197221

[5] TuMMLeeFJonesRTKimballAKSaraviaEGrazianoRF. Targeting DDR2 enhances tumor response to anti-PD-1 immunotherapy. Sci Adv (2019) 5(2):v2437. doi: 10.1126/sciadv.aav2437 PMC638240130801016

[6] ParkWChawlaAO'ReillyEM. Pancreatic cancer: A review. JAMA (2021) 326(9):851–62. doi: 10.1001/jama.2021.13027 PMC936315234547082

[7] HeYSiebuhrASBrandt-HansenNUWangJSuDZhengQ. Type X collagen levels are elevated in serum from human osteoarthritis patients and associated with biomarkers of cartilage degradation and inflammation. BMC Musculoskelet Disord (2014) 15:309. doi: 10.1186/1471-2474-15-309 25245039PMC4179849

[8] MäkitieOSusicMWardLBarclayCGlorieuxFHColeWG. Schmid type of metaphyseal chondrodysplasia and COL10A1 mutations–findings in 10 patients. Am J Med Genet A (2005) 137A(3):241–8. doi: 10.1002/ajmg.a.30855 16088909

[9] ShenG. The role of type X collagen in facilitating and regulating endochondral ossification of articular cartilage. Orthod Craniofac Res (2005) 8(1):11–7. doi: 10.1111/j.1601-6343.2004.00308.x 15667640

[10] CoghlanRFOberdorfJASienkoSAionaMDBostonBAConnellyKJ. A degradation fragment of type X collagen is a real-time marker for bone growth velocity. Sci Transl Med (2017) 9(419). doi: 10.1126/scitranslmed.aan4669 PMC651619429212713

[11] SoléXCrous-BouMCorderoDOlivaresDGuinóESanz-PamplonaR. Discovery and validation of new potential biomarkers for early detection of colon cancer. PloS One (2014) 9(9):e106748. 10.1371/journal.pone.01067482521550610.1371/journal.pone.0106748PMC4162553

[12] KaragozKLehmanHLStairsDBSinhaRArgaKY.. Proteomic and metabolic signatures of esophageal squamous cell carcinoma. Curr Cancer Drug Targets (2016).26845434

RETRACTED

[13] LiTHuangHShiGZhaoLLiTZhangZ. TGF-β1-SOX9 axis-inducible COL10A1 promotes invasion and metastasis in gastric cancer *via* epithelial-to-mesenchymal transition. Cell Death Dis (2018) 9(9):849. doi: 10.1038/s41419-018-0877-2 30154451PMC6113209

[14] BrodskyASXiongJYangDSchorlCFentonMAGravesTA. Identification of stromal ColXα1 and tumor-infiltrating lymphocytes as putative predictive markers of neoadjuvant therapy in estrogen receptor-positive/HER2-positive breast cancer. BMC Cancer (2016) 16:274. doi: 10.1186/s12885-016-2302-5 27090210PMC4835834

[15] ChapmanKBPrendesMJSternbergHKiddJLFunkWDWagnerJ. COL10A1 expression is elevated in diverse solid tumor types and is associated with tumor vasculature. Future Oncol (2012) 8(8):1031–40. doi: 10.2217/fon.12.79 22894674

[16] HuangHLiTYeGZhaoLZhangZMoD. High expression of COL10A1 is associated with poor prognosis in colorectal cancer. Onco Targets Ther (2018) 11:1571–81. doi: 10.2147/OTT.S160196 PMC586556529593423

[17] LiuQZhaoHGuoYZhangKShangFLiuT. Bioinformatics-based analysis: Noncoding RNA-mediated COL10A1 is associated with poor prognosis and immune cell infiltration in pancreatic cancer. J Healthc Eng (2022) 2022:7904982. doi: 10.1155/2022/7904982 36105715PMC9467764

[18] FavreauAJVaryCPBrooksPCSathyanarayanaP.. Cryptic collagen IV promotes cell migration and adhesion in myeloid leukemia. Cancer Med (2014) 3(2):265–72. doi: 10.1002/cam4.203 PMC398707624519883

[19] WangYZhangTGuoLRenTYangY.. Stromal extracellular matrix is a microenvironmental cue promoting resistance to EGFR tyrosine kinase inhibitors in lung cancer cells. Int J Biochem Cell Biol (2019) 106:96–106. doi: 10.1016/j.biocel.2018.11.001 30471423

[20] WuXCaiJZuoZLiJ. Collagen facilitates the colorectal cancer stemness and metastasis through an integrin/PI3K/AKT/Snail signaling pathway. BioMed Pharmacother (2019) 114:108708. doi: 10.1016/j.biopha.2019.108708 30913493

[21] ShenYShenRGeLZhuQLiF. Fibrillar type I collagen matrices enhance metastasis/invasion of ovarian epithelial cancer *via* β1 integrin and PTEN signals. Int J Gynecol Cancer (2012) 22(8):1316–24. doi: 10.1097/IGC.0b013e318263ef34 23013730

[22] RammalHSabyCMagnienKVan-GulickLGarnotelRBuacheE. Discoidin domain receptors: Potential actors and targets in cancer. Front Pharmacol (2016) 7:55. doi: 10.3389/fphar.2016.00055 27014069PMC4789497

[23] HuangHSvobodaRALazenbyAJSaowapaJChaikaNDingK. Up-regulation of n-cadherin by collagen I-activated discoidin domain receptor 1 in pancreatic cancer requires the adaptor molecule Shc1. J Biol Chem (2016) 291(44):23208–23. doi: 10.1074/jbc.M116.740605 PMC508773827605668

RETRACTED

[24] IwaiLKPayneLSLuczynskiMTChangFXuHClintonRW. Phosphoproteomics of collagen receptor networks reveals SHP-2 phosphorylation downstream of wild-type DDR2 and its lung cancer mutants. Biochem J (2013) 454(3):501–13. doi: 10.1042/BJ20121750 PMC389379723822953

[25] RadaMNallanthighalSChaJRyanKSageJEldredC. Inhibitor of apoptosis proteins (IAPs) mediate collagen type XI alpha 1-driven cisplatin resistance in ovarian cancer. Oncogene (2018) 37(35):4809–20. doi: 10.1038/s41388-018-0297-x 29769618

[26] LeitingerBKwanAP. The discoidin domain receptor DDR2 is a receptor for type X collagen. Matrix Biol (2006) 25(6):355–64. doi: 10.1016/j.matbio.2006.05.006 16806867

[27] ValiathanRRMarcoMLeitingerBKleerCGFridmanR.. Discoidin domain receptor tyrosine kinases: new players in cancer progression. Cancer Metastasis Rev (2012) 31(1-2):295–321. doi: 10.1007/s10555-012-9346-z 22366781PMC3351584

[28] XieBLinWYeJWangXZhangBXiongS. DDR2 facilitates hepatocellular carcinoma invasion and metastasis *via* activating ERK signaling and stabilizing SNAIL1. J Exp Clin Cancer Res (2015) 34(1):101. doi: 10.1186/s13046-015-0218-6 26362312PMC4567819

[29] LiangZXieWJZhaoMChengGPWuMJ.. DDR2 facilitates papillary thyroid carcinoma epithelial mesenchymal transition by activating ERK2/Snail1 pathway. Oncol Lett (2017) 14(6):8114–21. doi: 10.3892/ol.2017.7250 PMC572761629250189

[30] JollyLANovitskiySOwensPMassollNChengNFangW. Fibroblast-mediated collagen remodeling within the tumor microenvironment facilitates progression of thyroid cancers driven by BrafV600E and pten loss. Cancer Res (2016) 76(7):1804–13. doi: 10.1158/0008-5472.CAN-15-2351 PMC487333926818109

[31] QiuSDengLLiaoXNieLQiFJinK. Tumor-associated macrophages promote bladder tumor growth through PI3K/AKT signal induced by collagen. Cancer Sci (2019) 110(7):2110–8. doi: 10.1111/cas.14078 PMC660980031120174

[32] XuSXuHWangWLiSLiHLiT. The role of collagen in cancer: from bench to bedside. J Transl Med (2019) 17(1):309. doi: 10.1186/s12967-019-2058-1 31521169PMC6744664

[33] RenTZhangJZhangJLiuXYaoL. Increased expression of discoidin domain receptor 2 (DDR2): a novel independent prognostic marker of worse outcome in breast cancer patients. Med Oncol (2013) 30(1):397. doi: 10.1007/s12032-012-0397-3 23307244

[34] ElkamhawyALuQNadaHWooJQuanGLeeK. The journey of DDR1 and DDR2 kinase inhibitors as rising stars in the fight against cancer. Int J Mol Sci (2021) 22(12). doi: 10.3390/ijms22126535 PMC823533934207360

[35] XuJLuWZhangSZhuCRenTZhuT. Overexpression of DDR2 contributes to cell invasion and migration in head and neck squamous cell carcinoma. Cancer Biol Ther (2014) 15(5):612–22. doi: 10.4161/cbt.28181 PMC402608424556606

RETRACTED

[36] CarafoliFHohenesterE. Collagen recognition and transmembrane signalling by discoidin domain receptors. Biochim Biophys Acta (2013) 1834(10):2187–94. doi: 10.1016/j.bbapap.2012.10.014 PMC433241423128141

[37] ShrivastavaARadziejewskiCCampbellEKovacLMcGlynnMRyanTE. An orphan receptor tyrosine kinase family whose members serve as nonintegrin collagen receptors. Mol Cell (1997) 1(1):25–34. doi: 10.1016/S1097-2765(00)80004-0 9659900

[38] VogelWFAbdulhusseinRFordCE. Sensing extracellular matrix: an update on discoidin domain receptor function. Cell Signal (2006) 18(8):1108–16. doi: 10.1016/j.cellsig.2006.02.012 16626936

[39] CorsaCABrenotAGritherWRVan HoveSLozaAJZhangK. The action of discoidin domain receptor 2 in basal tumor cells and stromal cancer-associated fibroblasts is critical for breast cancer metastasis. Cell Rep (2016) 15(11):2510–23. doi: 10.1016/j.celrep.2016.05.033 PMC490954027264173

[40] WangZLFanZQJiangHDQuJM. Selective cox-2 inhibitor celecoxib induces epithelial-mesenchymal transition in human lung cancer cells *via* activating MEK-ERK signaling. Carcinogenesis (2013) 34(3):638–46. doi: 10.1093/carcin/bgs367 23172668

[41] ZhengFWuJZhaoSLuoQTangQYangL. Baicalein increases the expression and reciprocal interplay of RUNX3 and FOXO3a through crosstalk of AMPKα and MEK/ERK1/2 signaling pathways in human non-small cell lung cancer cells. J Exp Clin Cancer Res (2015) 34(1):41. doi: 10.1186/s13046-015-0160-7 25948105PMC4457308

[42] GaoYZhouJLiJ. Discoidin domain receptors orchestrate cancer progression: A focus on cancer therapies. Cancer Sci (2021) 112(3):962–9. doi: 10.1111/cas.14789 PMC793577433377205

[43] TeraiHTanLBeauchampEMHatcherJMLiuQMeyersonM. Characterization of DDR2 inhibitors for the treatment of DDR2 mutated nonsmall cell lung cancer. ACS Chem Biol (2015) 10(12):2687–96. doi: 10.1021/acschembio.5b00655 PMC468594326390252

[44] ZhangKCorsaCAPonikSMPriorJLPiwnica-WormsDEliceiriKW. The collagen receptor discoidin domain receptor 2 stabilizes SNAIL1 to facilitate breast cancer metastasis. Nat Cell Biol (2013) 15(6):677–87. doi: 10.1038/ncb2743 PMC379471023644467

[45] HammermanPSSosPSRamosMLXuAHDuttCZhouAW. Mutations in the DDR2 kinase gene identify a novel therapeutic target in squamous cell lung cancer. Cancer Discov (2011) 1(1):78–89. doi: 10.1158/2159-8274.CD-11-0005 22328973PMC3274752

[46] LeitingerB. Discoidin domain receptor functions in physiological and pathological conditions. Int Rev Cell Mol Biol (2014) 310:39–87. doi: 10.1016/B978-0-12-800180-6.00002-5 24725424PMC4021107

